RETRACTED

# MuTraff: A Smart-City Multi-Map Traffic Routing Framework

**DOI:** 10.3390/s19245342

**Published:** 2019-12-04

**Authors:** Alvaro Paricio, Miguel Angel Lopez-Carmona

**Affiliations:** Departamento de Automática, Campus Universitario Universidad de Alcala, Ctra. Madrid-Barcelona, km. 33.600, Alcalá de Henares, 28805 Madrid, Spain; miguelangel.lopez@uah.es

**Keywords:** intelligent transportation systems, dynamic traffic assignment, gas emissions, traffic management systems, traffic simulation, vehicle routing, smart cities, traffic big data, urban computing, crowdsensing, multi-agent systems, multimap routing, TWM

## Abstract

Urban traffic routing is deemed to be a significant challenge in intelligent transportation systems. Existing implementations suffer from several intrinsic issues such as scalability in centralized systems, unnecessary complexity of mechanisms and communication in distributed systems, and lack of privacy. These imply force intensive computational tasks in the traffic control center, continuous communication in real-time with involved stakeholders which require drivers to reveal their location, origin, and destination of their trips. In this paper we present an innovative urban traffic routing framework and reference architecture (multimap traffic control architecture, MuTraff), which is based on the strategical generation and distribution of a set of traffic network maps (traffic weighted multimaps, TWM) to vehicle categories or fleets. Each map in a TWM map set has the same topology but a different distribution of link weights, which are computed by considering policies and constraints that may apply to different vehicle groups. MuTraff delivers a traffic management system (TMS), where a traffic control center generates and distributes maps, while routing computation is performed at the vehicles. We show how this balance between generation, distribution, and routing computation improves scalability, eases communication complexities, and solves former privacy issues. Our study presents case studies in a real city environment for (a) global congestion management using random maps; (b) congestion control on road incidents; and c) emergency fleets routing. We show that MuTraff is a promising foundation framework that is easy to deploy, and is compatible with other existing TMS frameworks.

## 1. Introduction

Efficient urban traffic routing is a key challenge in the development of modern intelligent transportation systems (ITS) for smart cities. Urban traffic routing is not only an issue of optimization of individual agent needs but also a problem of citizen wellness and an ecosystem of services with conflicting interests and regulation: individual mobility, multi-modal mobility, safety, noise footprints, pollution and gas emissions, restricted areas that are geo-fenced, time-bounded commercial distribution, city space for public event usage, special fleets management, public transportation, and others [1,2]. All these factors can provide a wide range of data sources and configure the urban computing environment, which ITS must handle to create effective solutions for urban mobility and transportation [3,4]. Urban computing is part of the smart city concept, conceived as the application of information and communication technologies (ICT) to enhance the quality and performance of the services provided to an urban area and its citizens [5,6].

RETRACTED

Traffic demand in urban environments involves diverse group demands that require multi-objective routing mechanisms [1,2]: the demand can be clustered by emissions labels and power sources [7,8], by their usage (public, taxi services, distribution routes, and shared or private trips), by time and date slots, and other considerations. Usually the “vehicle class” concept refers to physical features such as size, payload, consumption, and emissions, but does not take into account the real value and expectations of the group needs. For instance, public transportation requires predictability and time effectiveness; private cars require travel routes that are time sensitive; electric vehicles require charging awareness; school transportation requires adherence to school time frames; local distribution transportation requires different time-sensitive routes; high-emission vehicles require geo-location and tracking, and so on. All of them use the same network, the same traffic data and make similar decisions. If we provide simultaneous and differentiated maps we could create a more effective environment in terms of value fulfillment. ITS need to provide differentiated routes to cover multi-objective traffic requirements.

Algorithms that use shortest-path methods are used for optimal route calculation, but usually converge to common driving decisions and induce congestion, since the optimal shortest-paths prefer to use the best-rated edges [9]. They use travel-time as a weight function, so link-distances and (max) speeds determine the preferred optimal routes. Route diversification is a key element to deliver resources in an efficient way. Several mechanisms have been proposed to deal with it: Centralized ones use hyperpaths and K-shortest-hyperpath variations to obtain route diversification [10,11,12,13]. On the other hand, distributed mechanisms provide ad-hoc local routing based on vehicle-to-vehicle (V2V) and vehicle-to-infrastructure (V2I) communications but they assume high computing and ideal connectivity capabilities in the vehicles and the infrastructure [14,15,16].

RETRACTED

There are many approaches to the design of efficient ITS that are centralized and distributed. However, they still have important challenges to be solved: architectural complexity, high connectivity and communications load, real-time data flows, high computing resources, big-data integration, and security and privacy, among others [17].

Routing algorithms and ITS rely on the use of traffic network maps. But what would happen if drivers used several different maps for the same network, or event map layouts that get refreshed? They would always be up-to-date and would consistently mark the best-route selection and driving decisions. Moreover, this type of format would be compatible with many of the available ITS and traffic agents.

We present Traffic Weighted Multimaps (TWM) as an innovative static and dynamic traffic routing mechanism based on the usage of complementary cost maps for vehicle groups, which enables differentiated planning and control policies. A TWM is formed by several collections of weights that refer to the edges of a physical traffic network. Every weight collection in the TWM offers a view of the physical traffic network that may be used by a vehicle routing agent of a fleet or category. Moreover, a group may also use several maps in the TWM to disperse route assignment between its member agents. Several cost functions can be used for TWM generation, considering some of the mentioned routing concerns: group interests, current traffic status, historical data, policies and regulation, constraints, and time incidents. Adequate TWM design may satisfy the objective control policy by grouping individual routing decisions. TWM is complementary to other routing strategies as it simply provides new maps policies that may be merged into existing frameworks.

Our work proposes an innovative traffic management system (TMS) architecture, called multimap traffic control architecture (MuTraff), that is data-centric. It provides generation and distribution of TWM by means of a centralized framework, which may be used in centralized, distributed, and autonomous vehicle routing scenarios. MuTraff requires less computing resources as TWM can be pre-calculated based on traffic data (historical or real time), traffic policies, and fleet constraints. TWM maps can be generated at certain timestamps or can be event based. The calculation of the best-route for every trip is performed by optimization algorithms that are based on the distributed TWM, either in the back-end or in the agent side. In terms of solving fleet needs, TWM differs from other approaches because it proposes differentiated maps per fleet, complementary to other routing algorithms and traffic agents.

RETRACTED

In MuTraff, dynamic maps may be updated in real time depending on traffic conditions. Static maps are pre-configured maps that are applied for a period of time. The main advantage of static maps is that they are simple and stable if the traffic conditions are known in advance, and there is no significant deviation during their application.

MuTraff offers a good balance between computational load, communications, and optimal results retrieval, levering the search for best-routes at the network level, and also enabling for vehicles that can do their own route computation. TWM is compatible with distributed traffic routing approaches by sharing the generated maps for their usage. In the same way, MuTraff can also be easily adapted to a distributed approach where multiple instances of MuTraff may be allocated at road-side units providing local TWM weight maps for routing.

MuTraff framework has a modular design that enables integration with other traffic frameworks. It provides the MuTraff simulator (MTS) component, which has been used in our experiments and it enables microscopic traffic simulation based on Simulation for Urban Mobility (SUMO) simulator  [18].

The main contributions of this paper include: (1) Discussion of traffic weighted multimaps (TWM) as an efficient method for stochastic static and dynamic traffic routing; and (2) description of a reference open architecture proposal (MuTraff) for TWM generation and distribution. Both allow for a system that is simple, scalable, secure, and compatible with other existing systems and easily deployable. It also needs less computational and communication requirements than other current solutions.

The paper also shows: (a) How TWM usage helps to reduce traffic congestion in urban networks, even with basic random policies; (b) how TWM implementation improves some smart city transportation-related indicators such as air-pollution, noise-emissions, and energy usage; (c) the positive impact of TWM on individual mobility experience; (d) the effectiveness of TWM when applied to urban incidents as a technique to reroute traffic; and (e) how TWM is used to cover specific fleet requirements.

The paper is structured as follows: There is an initial review of the state-of-art and related works, followed by the introduction of the traffic weighted multimap proposal. Next, we introduce the architectural framework MuTraff that supports TWM, which is the main contribution of the paper. Three case studies are presented using a real traffic network (Alcala de Henares, Spain): (a) traffic congestion control through random TWM maps; (b) congestion management on traffic incidents, and (c) emergency fleets routing. We then expose the simulation results and analyze the impacts of TWM over main urban traffic management concerns: global mobility and congestion, pollution and emissions, noise footprint, and individual driving experience. Finally, we draw conclusions and future research lines on TWM.

RETRACTED

## 2. Related Works

We first presented the traffic weighted multimaps method in [19] as an introductory proof of concept for congestion mitigation, and  tested it on synthetic networks based on grid networks. It is based on a centralized TMS MuTraff (cloud) by receiving and processing traffic information, which is later distributed to the vehicles in traffic weighted multimaps.

There are many centralized TMS proposals that provide viable traffic routing management solutions, as we can see in [20,21,22,23]. Some of these TMS, like SCORPION, UCONDES and others, acquire and periodically process information about the network and the individuals, detect traffic conditions, and generate routes that are distributed to the vehicles. Traffic information is obtained via beacons that are emitted periodically by the vehicles. The TMS then processes the data received using an algorithm such as a neural network, evolutionary algorithm [24,25], anticipatory and negotiation [26], or others. Relevant traffic information is sent to the vehicles in the network, which must decide whether to follow their current route or compute an alternative route. These centralized TMS procedures can choke the network when there is a high density of vehicles, and  additional improvements need to be made to reduce the volume of necessary communications.

Many distributed TMS designs have also been proposed to solve the limitations of the centralized TMS [27,28,29] such as DIVERT. The observations and interactions at various vehicle traffic agents provides the core knowledge about traffic conditions and interactions. Distributed cooperative TMS do not require a specific infrastructure for congestion detection as they rely on vehicle interactions to compute routes [16,30,31]. However, in the case of having an inefficient information exchange between vehicles, distributed TMS may suffer from similar issues as the centralized methods. Souza [16,28] proposed opportunistic content sharing by sending local information to certain areas, limiting the amount of communications required in the same way that individual notifications need to be controlled in centralized approaches. It assumes that critical sections are known in advance to limit those communications, being implicit the existence of a centralized TMS. V2I based mechanisms were also proposed in [15] but they have similar constraints as distributed TMS.

RETRACTED

An effective implementation of distributed routing requires that all the vehicles in the network have corresponding routing agents installed and running. Vehicle software agents should be available regardless of the vehicle fleet or class (cars, taxis, buses, trucks, vans, etc), and also should be vendor-neutral to assure cross-compatibility. Global adoption of distributed agent-based methods need an industry-wide consensus and would need the adoption of standards across the board, unless they are are capable of demonstrating their effectiveness under low-adoption scenarios. Another important drawback on distributed TMS is that they rely heavily on communications and permanent connectivity, which in turn depends on many factors: real vehicle communications capabilities, radio network properties including weather effects (such as fading), service providers, connectivity offerings, and subscription plans.

The hyperpath routing approach addresses uncertainty and variability of traffic dynamics, where individual traffic agents receive for each origin and destination a tree of alternatives, as opposed to a single route [10,11,13,32]. It feeds off historical data to discern traffic behavior patterns [12,33,34], thus requiring heavy back-end computing to synthesize the pre-trips. TWM is complementary to hyperpaths as it provides different network views for hyperpath calculation.

Urban traffic management using TMS with big-data approaches has been the subject of intensive research already, leading to proposals that differ in the way they implement traffic control and recommendations [35,36]. They are a core part of the smart city infrastructure approach that focuses on global parameters and specific fleet needs [37,38,39,40,41]. Big-data back-ends require real data-sets that are achieved using network sensors and crowdsensing approaches, where both the vehicle agent and the driver agent anonymously collect data from traffic and network status [42,43,44,45,46].

User-equilibrium in traffic flows is described by [47] and has been addressed by traffic routing approaches based on route aggregations as described by [48]. Aggregation also includes traffic routing based on static or dynamic flow exchange between areas (traffic assignment zones, TAZ) [49,50].

TWM is multi-purpose and combines individual, group, and global policies, in contrast to other centralized proposals that are conceived for individual risk-averse policies (minimizing travel-time variance). TWM is a stochastic routing technique, and thus optimal theoretical solutions are not achieved in comparison with other centralized solutions. Instead, TWM is a feasible, compatible, and easily deployable solution.

RETRACTED

## 3. Traffic Weighted Multimaps

This section provides the TWM model formulation and explains map generation strategies. Table 1 summarizes the model formulation.

### 3.1. TWM Model Formulation

The topological traffic representation of the urban network Θ, is described by a graph of nodes $\eta_{n}$ connected by unidirectional edges, being each edge $\epsilon_{i,j}$ a set of links (lanes) that connects nodes $\eta_{i}$ and $\eta_{j}$ with a weight $\beta_{i,j}$ as expressed by Equation (1). Edge travel-time is commonly used to estimate weight $\beta_{i,j}$ to compute shortest-path calculations.

(1) $$\Theta =\left\{\left[\eta_{n}\right],\left[\epsilon_{i,j}\right]\right\},\;\epsilon_{i,j}=\left(\eta_{i},\eta_{j},\beta_{i,j}\right).$$

The traffic network is commonly used by *k* groups of vehicles $\left[\Omega_{k}\right]$ that differ in their mobility features, objectives, and interests. Vehicles are represented by their agents $\left[\upsilon_{a}^{k}\right]$, where *a* denotes individuals belonging to the traffic demands of $\left[\Omega_{k}\right]$. The default fleet for non-grouped vehicles is $\Omega_{0}$.

Agents $\left[\upsilon_{a}^{k}\right]$ move in the traffic network generating a set of trips $\left[W_{a}^{k}\right]$, which are individually defined by the vehicle identification $\upsilon_{a}^{k}$, the starting timestamp $t_{a}^{0}$, the starting node $O_{a}$, the  destination node $D_{a}$, and the set of intermediate planned stops $[P_{a}^{k}]:$

(2) $$\begin{array}{c} W_{a}^{k}=f\left(\upsilon_{a}^{k},t_{a}^{0},O_{a},D_{a},\left[P_{a}^{k}\right]\right)\;\forall \upsilon_{a}^{k}\in \Omega_{k}. \end{array}$$

We define a multi map TWM, denoted by $\left[\mu_{k,m}\right]$, as the collection of *m* weighted views (maps) of the traffic network Θ, which can be used by the *k* traffic groups that use it.

Each map $\mu_{k,m}$ is as a edge weighted $\left[\beta_{i,j}^{k,m}\right]$ representation of the traffic network Θ (view k,m), which is calculated as the result of applying a function Π over (a) the network topology; (b) traffic groups or fleets $\left[\Omega_{k}\right]$; (c) time-constraints $\left[\Gamma_{k,m}\right]$ for usage; and (d) network traffic data Φ.

(3) $$\Pi :\Theta ,\left[\Omega_{k}\right],\left[\Gamma_{k,m}\right],\Phi \to \left[\mu_{k.m}\right],\;\mu_{k,m}=\left\{\left[\epsilon_{i,j}\right],\left[\beta_{i,j}^{k,m}\right],\Gamma_{k,m}\right\}.$$

Time constraints $\left[\Gamma_{k,m}\right]$ consider both periodic scheduled constraints (e.g., based on traffic restrictions, and school paths) and event-based time constraints (e.g., road works, public events, and road incidents).

RETRACTED

### 3.2. TWM Generation Policies for Traffic Planning

TWM generation policies are based on two main factors: (a) weight generation functions Π, and (b) map cardinality *m*. The latter enables that every fleet may use several maps at the same time. We use this parameter to provide route dispersion required for global congestion management. Map cardinality *m* is a design parameter. It may be part of TWM optimization algorithms planned for future works.

Different strategies may be applied for Π: linear scaling, random distributions, predictions over historical data, optimization functions, genetic algorithms, and others. In this paper we cover basic linear and random functions, leaving the rest for future works. The basic linear scaling function $\Pi_{std}$ (standard function), generates TWM weights based on scaling edge minimum travel-time $tt_{i,j}$ by a constant factor $k_{1}$. Weight scaling with $\Pi_{std}$ may be used to encourage ($k_{1}>1$) or discourage ($k_{1}<1$) usage of edges:

(4) $$\Pi_{std}:{\left[\epsilon_{i,j}\right]}_{A},\left[\Omega_{k}\right],\left[\Gamma_{k,m}\right]\to \left[\mu_{k.m}\right]\;|\;\beta_{i,j}^{k,m}=k_{1}*tt_{i,j}.$$

In the incident management scenario we need to over-weight part of the network around the incident to discourage vehicles from using that surrounding area. Adjacent edges may have very different original weights and the scaling factor $k_{1}$ is not enough to exclude some edges from the shortest-paths. This is best achieved using an additive factor $k_{2}$ as expressed by the linear function $\Pi_{lin}$ Equation (5). $\Pi_{lin}$ is useful for dynamic traffic routing applying local penalties or incentives:

(5) $$\Pi_{lin}:{\left[\epsilon_{i,j}\right]}_{A},\left[\Omega_{k}\right],\left[\Gamma_{k,m}\right],R_{x}\to \left[\mu_{k.m}\right]\;|\;\beta_{i,j}^{k,m}=k_{1}*tt_{i,j}+k_{2}.$$

In the global congestion management scenario, we need for similar trips to select slightly different shortest-path routes. Similar trips are those used by vehicles of the same fleet moving from the same origin TAZ to the same destination TAZ. This is accomplished distributing randomized maps to the vehicles of the same fleet. We use the $\Pi_{\delta }$ random function that modifies the $\Pi_{std}$ function with a random modifier δ:

(6) $$\Pi_{\delta }:\left[\epsilon_{i,j}\right],\left[\Omega_{k}\right],\left[\Gamma_{k,m}\right]\to \left[\mu_{k.m}\right]\;|\;\beta_{i,j}^{k,m}=k_{1}*tt_{i,j}*\left(1+\delta \right).$$

Routing decisions using TWM with $\Pi_{\delta }$ are going to disperse traffic in the network as shortest-paths will vary their composition. The aim of TWM is to stochastically route groups of vehicles through specific network links in a one-shot fashion by generating maps with different link weights. Initial reference weights that generate different maps are defined in terms of delay for free-flow. Of course, other strategies for generating link weights offline could be based on using volume delay functions and dynamic traffic assignment for traffic prediction.

RETRACTED

We use $\Pi_{\delta }$ random in our experiments with normal and uniform distributions using δ as $\delta_{normal}=normal\left(a,b\right)$ (*a* stands for the mean value and *b* stands for the statistical dispersion amplitude) and $\delta_{uniform}=uniform\left(a,b\right)$ (ranging from *a* to *b*).

### 3.3. TWM for Urban Traffic Routing

Not all the agents will use TWM so we define the adherence factor ψ in Equation (7) as the percentage of agents ${\left[\upsilon_{a}^{k}\right]}_{TWM}$ that are using it. We use ψ to compare different TWM adoption scenarios.

(7) $$\psi =\frac{\sum {\left[\upsilon_{a}^{k}\right]}_{TWM}}{\sum \left[\upsilon_{a}^{k}\right]}.$$

Agents belonging to $\Omega_{0}$ fleet (non-classified vehicles) and agents not adhering to TWM use the map $\mu_{0}$ with $\beta_{i,j}^{0}=tt_{i,j}$ that corresponds to the original physical map.

Independently of client or server routing modes, the routing agent $\upsilon_{a}^{k}$ calculates the best route $R_{a}^{k,m}$ in Equation (8) or hyperpath for the trip $W_{a}^{k}$, using the physical map $\mu_{0}$ or the TWM $\mu_{k,m}$. Best-route calculation algorithms *⨙* can be used for this, such as Dijkstra, A* or others:

(8) $$R_{a}^{k,m}=\left\{\begin{array}{cc} \left(⨙O_{i},D_{a}^{k},\left[P_{a}\right],\mu_{k,m}\right) & \upsilon_{a}^{k}\in {\left[\upsilon_{a}^{k}\right]}_{TWM}\\ \left(⨙O_{i},D_{a}^{k},\left[P_{a}\right],\mu_{0}\right) & \upsilon_{a}^{k}\notin {\left[\upsilon_{a}^{k}\right]}_{TWM} \end{array}\right..$$

Total travel-time $TT_{a}^{k}$ of a mobile agent $\upsilon_{a}^{k}$ is composed of congested $STT_{a}^{k}$ and non-congested $MTT_{a}^{k}$ travel-times, as the sum of the partial travel-times at each edge, Equation (9). $\sum STT_{a}^{k}$ provides a good measure of global congestion in the traffic network.

(9) $$TT_{a}^{k}=STT{}_{a}^{k}+MTT_{a}^{k}.$$

Effective trip length $RL_{a}^{k}$ run by an agent is the sum of lengths of every edge:

(10) $$RL_{a}^{k}=\sum length\left(\epsilon_{i,j}\right),\epsilon_{i,j}\in R_{a}^{k,m}.$$

For traffic routing performance analysis, we consider at every timestamp *t* those trips that have been already completed ${\left[W_{a}^{k}\right]}_{end}^{t}$, those that have been started ${\left[W_{a}^{k}\right]}_{run}^{t}$ and not completed ${\left[W_{a}^{k}\right]}_{pend}^{t}$, and  those that have not been started yet (Equation (11)):

(11) $${\left[W_{a}^{k}\right]}_{total}^{t}={\left[W_{a}^{k}\right]}_{end}^{t}\cup {\left[W_{a}^{k}\right]}_{run}^{t}\cup {\left[W_{a}^{k}\right]}_{pend}^{t}.$$

RETRACTED

## 4. MuTraff Architecture

Multimap traffic management requires a specific architecture approach for a feasible physical deployment. In this paper we propose a full-stack reference architecture called MuTraff (Multimap Traffic Control Architecture) that may be used as stand-alone system or combined with already existing traffic architectures.

From the perspective of a vehicle’s agent, *MuTraff* may be considered as a TWM-based routing service provider that offers custom traffic network maps services, and also efficient origin-destination routing services. From the perspective of the traffic service operator, *MuTraff* can be considered as a low-impact traffic analysis and optimization tool and a traffic big-data processor.

One of the main objectives of *MuTraff* is to provide a set of components that integrate seamlessly with current systems by means of standard interfaces, being also compatible with standard traffic agents software. Some of the reference blocks may be provided by existing traffic management frameworks, devices and tools, but some others are new elements added to cover the TWM algorithms and functionality.

Part of the building blocks are already available and others are under construction or in the backlog. Experiment results shown in the paper have been obtained with these blocks. *MuTraff* main blocks (modules) are shown in Figure 1:

- *MuTraff big-data core (MDB)*. It collects data from the different sources available: historical traffic data, traffic planning data, and real-time dynamics monitoring. Historical sources considered are:
  - Traffic demands (from road sensing), both aggregated and per fleet when available.
  - Edge measures for traffic density, speed and congestion, pollution measures, and noise emissions. These measures are collected from many different sources such as road sensors, vehicle sensors, crowdsensing, and others.
  - Individual historical traffic demands that have been collected from the vehicle mobile agents through crowdsensing mechanisms regarding origin/destination trips and frequencies, and also from back-office routing services. Agents also report information about speeds.
  - Driver experience historical information about map demands, satisfaction, engagement, and others.
  Planning data reflects traffic behaviors detected under certain past situations that enable model and pattern detection. Dynamic data are collected in a continuous way from the sensors and from the vehicle agents.
  The MuTraff Big-Data component will generate data predictions over each network path indicating traffic density, congestion, speeds, pollution, emissions, and user-experience. It mainly calculates in several time-epochs the weight distribution functions Π for the different traffic networks $\left[\Theta_{i}\right]$. This Big-Data module uses a data-lake approach ([51,52,53]) to collect data, and may use a machine-learning subsystem to detect traffic patterns and infer the corresponding weights for Π.
- *MuTraff central control station (MCCS)*. The purpose of this component is to generate traffic weighted maps $\left[\mu_{k,m}\right]$ according to the data collected from the big-data module and from the real-time sensor data. Its main module is the MuTraff map manager (MTMapManager) for TWM generation, management and distribution.
  The MCCS provides two main families of services for traffic agents, provided as web services:
  - *Map services*, for TWM generation and distribution under several policies (broadcast, publish-subscribe, and on-demand). These services are designed to be used at agent-side route calculation.
  - *Route services,* for querying origin/destination routes or hyperpaths based on server-side TWM maps. These services are used when the agent asks for a route from origin to destination.
  MCCS is not intended to be provided as a full featured control station, but to serve as a plugin for other control stations. The MCCS includes all the necessary algorithms for weighted maps generation and also the route generation procedures for individual origin-destination trips. The MCCS is conceived to be offered as a cloud service, with  a web portal and a REST-API offering.
  If we recall Equation (3): $\Pi :\Theta ,\left[\Omega_{k}\right],\left[\Gamma_{k,m}\right],\Phi \to \left[\mu_{k.m}\right]$, TWM depends on the traffic area (city), group of fleets, time-constraints, and traffic events. There is no need to recalculate the TWM for every agent call, but just when any of these parameters change. MCCS caches the $\left[\mu_{k.m}\right]$ map to provide fast responses to the agents.
- *MuTraff data distribution middleware (DMW)*. This component enables distributed communications between all the components, and  mainly between traffic agents and the MCCS, decoupling core engines from the consuming agents, creating an loosely-coupled and scalable architecture. It is a distributed cloud for server-side middleware that exposes and manages services as APIs using different policies (REST, Pub-sub, and others). Sensors and actuators use both web-services and publish-subscribe real-time queue oriented communications. Agents, sensors and actuators are not part of the middleware using just secured services in the framework.
- *Sensor and actuator network (SAN)*. These sensor and actuator networks include the common standard traffic measurement and signaling systems. We consider two kinds of sensors: physical sensors and crowdsensing devices to acquire real-time data about the network, traffic status, and driver’s behavior. They provide the necessary information to create dynamic traffic assignment, and also provide information about driver’s adherence to TWM recommendations.
- *Mobile traffic agents (MTA)*. Traffic agents are standard navigation software agents. From the route calculation mode perspective, there are three main types of mobile traffic agents: (a) online agents, that require a permanent active data-connection to ask for the best route sets during their trips, (b) autonomous agents that just download the traffic maps and the status information, that execute their own client-side route calculation, and (c) hybrid agents using a download basis that is periodically updated by online real-time data. The MCCS provides TWM services for all of them.
- *MuTraff traffic simulator (MTS)*, that enables traffic simulation and route evaluations based on TWM maps before they are deployed to real traffic. Generated TWM maps may also be used with almost any of the standard simulation platforms as they act over standard common variables, such as traffic demands per fleet and network maps. Network maps are a key data entry for any existing traffic simulator, so TWM approach is valid for microscopic, mesoscopic, and macroscopic simulators as they all use the network as a basis.
  Current simulations presented in this paper have been run on MTS over the well known SUMO traffic microscopic car-following simulator [18]. MTS manages traffic simulation based on vehicle traffic demands, physical road maps, and colored-weighted maps produced from the MCCS. The simulator can be run with the graphical interface typically available for SUMO where individual vehicles are shown over time, but also as a multi-threaded distributed process that scales horizontally. MTS also generates the traffic indicators mentioned in the model formulation Section 3.1.
- *MuTraff traffic and maps toolbox (MTools)*. New auxiliary tools are being constantly added to the platform to provide additional capabilities to manage and administer data and for simulation purposes. Some of them are:
  - *MuTraff TAZ Designer (MTTaz)* that provides a web interface for easy graphic ttraffic assignment zones (TAZ) generation and management.
  - *MuTraff Origin/Destination (O/D) matrix Traffic Matrix Generator (MTodMatrix)* for O/D synthesis with traffic distributions in time.
  - *MuTraff Map Converter (MTMapConverter)* for map translation.
  - *MuTraff Traffic Demand Generator (MTDemandGen)* for traffic demand generation with certain statistical distributions.
  - *MuTraff Reporting Engine* for TWM traffic impact analysis.

RETRACTED

In Figure 2 we zoom into the building blocks of the server-side components: MCCS, MDB, MTS, and DWM. Also SAN is included for completion purposes.

### 4.1. The MCCS Control Station

The MCCS is a server-side service used to generate Traffic Weighted Maps (TWM $\left[\mu_{k,m}\right]$) according to the data collected from the big-data module and from the real-time sensor data. It is formed by the following architectural modules:

- The *MuTraff map manager (MTMapManager)* in charge of TWM generation, management and distribution based on statistical information. It is responsible for evaluating the $\Pi_{x}$ functions for each network Θ, and generating $\left[\mu_{k,m}\right]$ for every time epoch.
- The *MuTraff route manager* is the module responsible for providing the query-based route or multi-path selection for agents (server-side) for those schemes where the agent sends a query for its trip $W_{a}^{k}$ and receives the corresponding $R_{a}^{k,m}$ route or hyperpath $\left[R_{a}^{k,m}\right]$.
- The *MuTraff BDI (Belief-Desire-Intentions) processor*, which is in charge of processing dynamic route demands to predict future traffic trends. This module is part of future work.
- The *MuTraff AlertManager*, responsible for publishing traffic alerts that will reinforce TWM adoption. These alerts are to be exposed both in the signaling panels and also in the mobile agents, promoting route re-evaluation with new TWM sets.
- The *MuTraff device network management*, responsible for sensors and actuators management, receiving from and sending data to them.

In its simplest form of operation, generation of maps in MuTraff is made in open loop, without feedback from vehicles or network. TWM maps can be generated considering historical traffic flow data or just applying traffic policies or recommendations. In this case it is not necessary for vehicles or sensors to send data to MuTraff. Consider, for instance, a traffic flow between a densely populated residential area and several educational centers located at a short distance between them. This flow can be known through manual counting, sensor counting, or crowdsourcing. In any of these cases, we may assume that data is obtained offline. This way, the path or paths of the flow can be estimated, and MuTraff will be able to apply a map generation algorithm based of these paths and flows. In addition, we may add dynamic traffic restriction policies for school entrance and exit times.

RETRACTED

In a scenario in which maps are generated in real-time depending on traffic conditions, counting is done in real time by means of sensors or crowdsourcing. In the case of using sensors, communication latency is not as critical as in the case of crowdsourcing because the number of sensors is significantly lower, and sensor data updates are usually in the order of minutes. In addition, current proposals in the mobile edge computing field would allow distribution of the computational load when estimating traffic flows in a distributed way. Only essential information of flows would be transmitted to MuTraff to generate maps.

In the case of failure in data sensor collection, the most straightforward recovery approach is to switch to open-loop mode (historic based map ‘static’ generation). However, the most appropriate system response will depend on the specific scenario.

### 4.2. The MDB Data Analyzer

The MDB data analyzer is the other core component in the architecture. It is used to do data-lake oriented processing and data clustering. Its main blocks are:

- The Traffic Demand Dissagregation unit, devoted to create synthetic statistical models of individual trips from the data collected from the path sensors in the traffic network.
- The Data-lake component oriented to collect raw-data in a log-oriented way, to create inferences from them.
- The Data Collection engine used to roughly parse data for injection into the data-lake.
- And the Traffic Predictor, which will generate distribution functions for the traffic network usage. They will be requested by the MCSS to generate the TWM maps. It is planned to use convolutional neural networks as those described by [54,55].

Dynamic origin destination estimation (DODE) [56] requires $\left[W_{a}^{k}\right]$ data as described in Equation (2). Extracting individual trips and flow data from the traffic link sensors is a non-trivial NP-Hard (non-deterministic polynomial-time hard) and time-dependent problem that requires high computation resources. It has been a subject of intense research for a long time and many approaches and models have been made [57,58,59]. But nevertheless, there are some direct ways of obtaining $\left[W_{a}^{k}\right]$ information: (a) cloud route calculation services that receive directly drivers requests; (b) tracing individual vehicles in the network (using cameras and other mechanisms); and (c) using crowdsensing mechanisms by means of a dedicated app or an embedded measurement rootkit in an app. This crowdsensing mechanism provides anonymous origin/destination trip data and the route taken, but only for a few vehicles. MuTraff MDB uses a combination of DODE model and crowdsensing direct data for contrast and validation.

RETRACTED

### 4.3. The MTS Simulation Engine

Traffic weighted maps $\left[\mu_{k,m}\right]$ may be used directly in current macro, meso, and microscopic traffic simulators, as they all use Θ network map representations. MuTraff implementation distributes either new network maps, or complementary-costs network maps that replace Θ maps for each individual or fleet.

Current MTS implementation uses SUMO, which implements a car-following microscopic simulation environment [9,18], perfectly fitting the proposed architecture. Figure 3 shows MTS main loop and SUMO integration.

### 4.4. The DMW Middleware

The DMW middleware layer offers the following interfaces for the agents (in REST-API mode):

- TWM distribution services, based on several models: (1) a downloadable network $\left[\mu_{k,m}\right]$ as a request for urban area Θ, and (2) a publication-subscribe notification interface for $\left[\mu_{k,m}\right]$ subscriptions on urban area Θ. This TWM service is used for client-based route calculation and offline TWM usage.
- Route calculation services to provide on-demand O/D routes $R_{a}^{k,m}$ to the agents.
- Real-time traffic alert services, to be used by road-signaling systems. They are oriented to increase the adherence factor ψ that will produce better traffic distributions.
- Agent oriented interfaces that will increase the performance of traffic prediction algorithms. Information provided by the agents is used to create forecasts for weighting the Π functions:
  - A route interface where the agent queries in advance its routing intentions or queries about distance and travel-times.
  - A feedback interface where the agent scores its utility from using the routing proposal.

TWM formats are customizable, and can be delivered using several methods, both as complete network maps (in OpenStreet MAps (OSM) format, for instance) or just as edge-weight maps, much more reduced in size. Current experiments use SUMO/XML. Different XML tags and attributes are used to describe the destination of a given map and its choice probability.

Many different alternatives in real scenarios may arise with the purpose of sending maps from MuTraff to vehicles, and then selecting the right map in the vehicle. The most straightforward approach is to periodically deliver a message with the updated set of maps. This set is formed by subsets of maps that we want to allocate to fleets or groups of vehicles (each subset to a fleet or group). We say ‘group’ of vehicles, because we may allocate TWM maps to vehicles attending other criteria than fleet belonging (i.e., ‘taxis’). For instance, we could allocate a specific map subset to vehicles located in a predetermined geographic area.

RETRACTED

Thus, each map subset in the message must be tagged at least with the ‘fleet’ or ‘group’ name, type, and corresponding options depending on type. A probability tag can be used for each map within the range of a subset, to define the choice probability of a map. For instance, a subset of 10 maps tagged with name = ‘residential A’, type = ‘area’, options = ‘x1, y1, x2, y2’, would define a subset that should be allocated to vehicles within geographical area (x1, y1, x2, y2). If for each map within the subset, the probability is defined as 0.1, each vehicle will select randomly any of the 10 maps with probability 0.1. The general idea is to define map descriptions (tags) to allow vehicles to filter maps.

To guarantee that different fleets or groups will only have access to their own maps, and that there is no disclosure of information, the most direct approach is to use https to guarantee server identity and send encrypted information. We assume that the navigation app in the vehicle protects received information from local disclosure. In the case of fleets (i.e., taxis and ambulances), vehicles will need to register the app to qualify themselves as belonging to a given fleet. In the case of maps that are tagged with geographical coordinates, the app will filter out depending on current GPS (global positioning system) vehicle position.

### 4.5. MuTraff Capabilities for Distributed Routing Environments

There is a broad consensus on the suitability of applying distributed routing techniques in connected and autonomous vehicle scenarios (CAV). The MuTraff architecture proposal is centralized from the perspective of creating and distributing maps, but the computational load for route calculation may be distributed. Thus TWM is not conceived categorically as a centralized system.

On the other hand, although MuTraff defines a single central station TMS that generates and distributes maps, it can be perfectly extended to a set of multiple distributed local stations (road-side units), with a bounded range of action that distributes local weights for routing. We can think of a scenario in which multiple local stations cooperate autonomously to generate maps that globally optimize traffic flows. TWM has applicability both in connected and autonomous vehicle environments, where vehicles may have the capacity to receive maps to decide their routes.

Cooperative behavior between vehicles when selecting routes is induced through strategic map generation, while in many other distributed routing systems, cooperation is performed at route level and not map level. Distributed solutions at vehicle-level may allow to compute optimal routes with a finer granularity, but with higher communication requirements. Using MuTraff, a vehicle only needs to receive maps through a broadcast channel. In distributed approaches, vehicles may need to communicate with other vehicles or with the infrastructure in bidirectional channels.

RETRACTED

### 4.6. MuTraff Technology and Practices

The MuTraff framework is based on open-source platforms in a modular style based on micro-services [60,61] enabling integration to third party tools. All the components run under light-weight docker containers using Linux [62,63,64], which allows platform agnostic deployments and on-premise or cloud deployments. Docker technology enables fast and simple micro-services adoption and distributed horizontal performance scaling.

Implementation technologies selected for the different components are:

- *MuTraff big-data core (MDB)*. There are many second generation big-data tools (improving the hive-hadoop reference) that provides the necessary capabilities. We selected *Apache Spark* [65,66] for the high performance and scalability of the solution.
- *MuTraff central control station (MCCS)*. This a web based traditional application written in python over a light-weight flask [67] web-server and mySQL database. The user interface is based on Google’s Angular [68].
- *MuTraff data distribution middleware (DMW)* is critical for decoupling the components of the framework and external integration. It is based on *Apache Kafka* [69,70,71] for advanced communications capabilities allowing consistent and flexible events streaming with high performance and *swagger* [72,73] as REST-API manager for micro-services exposure and integration.
- *MuTraff traffic simulator (MTS)* is a proprietary design in python to integrate with external traffic simulation engines. This paper uses SUMO Traci integration interface [74].
- *Mobile traffic agents (MTA)*. Any vehicle or personal routing agent supporting REST-API is able to be used, and adapter interfaces are easily developed. Specific MTA is still a work in progress.
- *Sensor and actuator network (SAN)*. Standard sensor networks may be integrated in the future by means of DWM. MTS provides SAN networks emulation.
- *MuTraff traffic and maps toolbox (MTools)*. Tools are scripted python components and analytic workbooks over jupyter-anaconda [75] for ease of use.

*MuTraff* also uses maps from OpenStreetMaps [76] and Amitran coding references [77].

## 5. Case Studies

The MuTraff framework has been tested with synthetic and real urban network topologies using traffic flows based on field demand measures. Tests have been carried out using MTS simulator.

RETRACTED

Several fleets have been considered for the case studies: cars, taxis, buses, and motorcycles with the distribution shown in Table 2. The *MTDemandGen* tool *(MuTraff Traffic Demand Generator)* and the SUMO tool *od2trips* have been used to create the end-user trips for the microscopic simulation. The same demand is used to compare no-TWM scenarios with the TWM application scenarios that use different driver adherences, different map number and configuration, and other parameters. Traffic is modeled using traffic assignment zones (TAZ) that are logical geo-fenced areas that contain interconnected nodes. TAZs are used to group sources and sinks of trips based on their origin and destination. Traffic demand is modeled with the set of flows between TAZs. There is no bulk demand uploading, as *MuTraff simulator MTS* injects every trip into the network in its specific timestamp. We consider a uniform distribution over time for all vehicles, as we use a single set of maps during the simulation period. In cases of 5-minute demand allocation, we could consider the calculation of maps every T minutes (T = 5, 10, or 15) and distribute them at once or allocate them temporarily. The maps that are assigned in the case studies have a certain temporal validity (temporal restriction), but  several sets of maps could be distributed or assigned selectively over time.

As well, the case studies consider several driver adherences to TWM: $\psi_{0.1}$, $\psi_{0.2}$, $\psi_{0.5}$, and $\psi_{1}$ as described in Table 3. For the emissions model we have used the HBEFA3 model described in  [7], which is available in the core simulation engine. Fleet emissions references are shown in Table 2. We start with a summary of TWM performance indicators that are to be considered. Then the real-urban network of Alcala de Henares is described, and  three scenarios of TWM application are evaluated: global traffic congestion reduction, mitigation of traffic congestion at road incidents and emergency fleets routing.

### 5.1. Global and Individual TWM Performance Indicators

In order to measure the wellness of TWM it is necessary to consider both global and individual impacts. Table 4 summarizes basic TWM indicators.

### 5.2. Global TWM Indicators

Global impacts in the traffic network consider congested edges, mean speed, total travel-times, pollution, noise, and some others:

- *$DTD^{t}$ dispatched traffic demand*, the percentage of routed demand compared against the total traffic demand exposed to the network:
  (12) $$DTD^{t}=\frac{card({\left[W_{a}^{k}\right]}_{end}^{t})}{card({\left[W_{a}^{k}\right]}_{total}^{t})}.$$
- $DTD_{TWM}$ *as successfully TWM routed traffic*, as  ratio of TWM routed traffic versus incoming traffic:
  (13) $$\begin{array}{cc} DTD_{TWM} & =\frac{card({\left[W_{a}^{k}\right]}_{TWM})}{card({\left[W_{a}^{k}\right]}_{total})}\;|\;W_{a}^{k}\in {\left[W_{a}^{k}\right]}_{end},\upsilon_{a}^{k}\in {\left[\upsilon_{a}^{k}\right]}_{TWM}. \end{array}$$
- *$TTS^{t}$ total time spent by the vehicles* in the traffic network:
  (14) $$TTS^{t}=\sum TT_{a}^{k}|W_{a}^{k}\in {\left[W_{a}^{k}\right]}_{end}^{t}\cup {\left[W_{a}^{k}\right]}_{run}^{t}.$$
- *$THS^{t}$, total halting time (congestion time, waiting time)*, as the total sum of halting times of the vehicles in the network:
  (15) $$THS^{t}=\sum STT_{a}^{k}|W_{a}^{k}\in {\left[W_{a}^{k}\right]}_{end}^{t}\cup {\left[W_{a}^{k}\right]}_{run}^{t}.$$
- *$NHD^{t}$ volume of halted demand (vehicles)* (minimum speed of 0.1 m/s):
  (16) $$\begin{array}{cc} NHD^{t} & =card\left(\left[v_{i}^{k}\right]\right)\;|\;W_{a}^{k}\in {\left[W_{a}^{k}\right]}_{end}^{t}\cup {\left[W_{a}^{k}\right]}_{run}^{t},\;speed\left(v_{i}^{k}\right)\leq \;0.1. \end{array}$$
- *VKT total distance traveled* by the vehicles that started their trips in the network:
  (17) $$VKT^{t}=\sum RL_{a}^{k}|W_{a}^{k}\in {\left[W_{a}^{k}\right]}_{end}^{t}\cup {\left[W_{a}^{k}\right]}_{run}^{t}.$$
- *$NMS^{t}$ network mean speed,* as mean speed of the running agents in an instant:
  (18) $$NMS^{t}=\sum s_{a}^{k}|W_{a}^{k}\in {\left[W_{a}^{k}\right]}_{run}^{t}.$$
- *$NMV^{t}$ number of active vehicles* in the network in an instant, with the variant of NMV(H) for number of halted vehicles:
  (19) $$NMV^{t}=count\left(v_{a}^{k}\right)|W_{a}^{k}\in {\left[W_{a}^{k}\right]}_{run}^{t}.$$
- *$NEO^{t}$ network edge occupancy* in the network in an instant, with the variant of NEO(C) for number of congested edges:
  (20) $$NEO^{t}=\sum ge_{a}^{k}|W_{a}^{k}\in {\left[W_{a}^{k}\right]}_{end}^{t}\cup {\left[W_{a}^{k}\right]}_{run}^{t}.$$
- *$GET_{NOx,CO,CO2,HC,PMx...}^{t}$ total gas emissions* produced by the routed vehicles:
  (21) $$GET^{t}=\sum ge_{a}^{k}|W_{a}^{k}\in {\left[W_{a}^{k}\right]}_{end}^{t}\cup {\left[W_{a}^{k}\right]}_{run}^{t}.$$
- *$NET^{t}$ total noise emissions* generated by the routed vehicles:
  (22) $$NET^{t}=\sum ne_{a}^{k}|W_{a}^{k}\in {\left[W_{a}^{k}\right]}_{end}^{t}\cup {\left[W_{a}^{k}\right]}_{run}^{t}.$$
- *$PCT_{Fuel,Electricity}^{t}$ total power consumption* used by the routed vehicles:
  (23) $$PCT^{t}=\sum pc_{a}^{k}|W_{a}^{k}\in {\left[W_{a}^{k}\right]}_{end}^{t}\cup {\left[W_{a}^{k}\right]}_{run}^{t}.$$

RETRACTED

### 5.3. Individual TWM Indicators

Individual impacts consider the user experience factors such as travel-time, trip cost, or route length. Individual concerns are critical for TWM as they influence driver confidence that is based on objective and subjective previous experiences, word-of-mouth experiences, social-media exposition and others. Individual impacts need to consider TWM users as well as non-TWM users.

To measure individual impacts we analyze the changes produced in every agent at the study variables when TWM is used compared to no TWM usage. Relative changes are considered together with paired statistics. The  variables under study are:

- $TTC_{rel}^{k}$ *Individual relative travel time change* (as a percentage over original travel-time), where $TT_{a}^{k}{¦}_{TWM}$ and $TT_{a}^{k}$ denote travel-time of a single trip using TWM or not respectively:
  (24) $${\mathrm{TTC}}_{\mathrm{rel}}^{k}=\frac{TT_{a}^{k}{¦}_{noTWM}-TT{}_{a}^{k}{¦}_{TWM}}{TT_{a}^{k}{¦}_{noTWM}}.$$
- *$RLC_{rel}^{k}$* *Individual route length relative change* (as a percentage over original route length), where $RL_{a}^{k}{¦}_{TWM}$ and $RL_{a}^{k}{¦}_{noTWM}$ denote route-length of a single trip using TWM or not respectively:
  (25) $$RLC_{rel}^{k}=\frac{RL_{a}^{k}{¦}_{noTWM}-RL_{a}^{k}{¦}_{TWM}}{RL_{a}^{k}{¦}_{noTWM}}.$$
- $MR_{a}^{k}$ *Individual motion rate* that helps us measure which time percentage of the individual trip routing is spent in vehicle motion (not halted):
  (26) $$MR_{a}^{k}=\frac{MTT_{a}^{k}}{TT_{a}^{k}}.$$

$MR_{a}^{k}$ provides a method to estimate individual experience when comparing two routing strategies $R_{1}$ and $R_{2}$, which have similar travel-times. $R_{1}$ has a better driving experience than other $R_{2}$ if $MR_{a}^{k}{¦}_{R_{1}}>MR_{a}^{k}{¦}_{R_{2}}$. Travel-times are said to be similar when their relative difference is bounded under a prefixed limit.

### 5.4. Urban Network Description

Alcala de Henares is a mid-size city with a population of 250,000 people, located 30 km north–east of Madrid, Spain. The city implements a wide variety of traffic scenarios as it is crossed by a main highway connecting Madrid and Barcelona that is used daily by thousands of private vehicles and light and heavy commercial distribution. The city has severe traffic restrictions and pedestrian areas due to the protected middle-age downtown and at the same time it contains many public citizen service facilities including part of the university campus. It also combines dense residential areas together with wide open residential ones. The city is surrounded by an industrial belt with many logistic companies established; the belt also contains wide commercial areas and also additional public facilities like hospitals and the rest of the campus. Alcala is very close to Madrid’s international airport and business centers, so there is a heavy daily traffic in and out mixing private, public and commercial traffic. It also has a heavy traffic exchange with close villages.

RETRACTED

### 5.5. TWM for Static Congestion Management

Our urban traffic network is split into traffic assignment zones (TAZ) in order to establish traffic flows, as shown in Figure 4 and Table 5. These flows are designed based on two data sources covering heavy traffic hours: (a) network sensor measures located in the main road connections; and (b) crowdsensing data obtained from ad-hoc mobile apps. The first data source enables synthetic flow calculation for the O/D matrix as it contains full traffic data but lacks trip O/D data; the second source provides real routes with O/D data and enables synthetic matrix validation. Figure 5 shows the position of vehicles and measures speed (blue for fast vehicles, red for slow ones). Only a small number of vehicles use the crowdsensing sdk-toolkit. Table 6 shows the TAZ traffic matrix for 2 h, where simulation covers an additional hour for traffic completion.

To obtain good results for static congestion management, we consider two objectives: traffic network usage maximized by vehicles routes, and trip travel-time minimized by means of best-route choice. This can be achieved using optimal distributions based on previous knowledge of real traffic demand or usage of historical data. This need can also be handled in a sub-optimal way by means of the TWM random function $\Pi_{\delta }$ Equation (6) with uniformly distributed weights around the edge speeds.

The case study uses a $\Pi_{\delta }$ TWM with 16 maps ($\mu_{1}$ to $\mu_{16}$), which are used by all the vehicles with the same probability as shown in Table 7. Map $\mu_{0}$ represent the original non-TWM network map that is used for the fixed routes for buses and also for the vehicles that do not adhere to TWM. They are not rerouted.

### 5.6. Ad-Hoc TWM for Incident Management

TWM may be used to reduce incident impact on global congestion. This incident may be planned or accidental. When an incident appears in the network it usually collapses the affected edge or node and the surrounding traffic area.

*MuTraff* is used to generate an ad-hoc TWM that modifies road weights around the incident edge ${\left[\epsilon {}_{i,j}\right]}_{x}$ with radius $R_{x}$ using $\Pi_{x}\to {\left[\mu_{k,m}\right]}_{x}$. It merges edge weights of the standard map $\mu_{0}$ or current $\left[\mu_{k,m}\right]$ if other TWM maps were being used. Radius selects the edges belonging to the feasible traffic paths of $card\left(Path_{i}\right)⪯R_{x}$ that converge to ${\left[\epsilon {}_{i,j}\right]}_{x}$. It is measured in number of edges as once the vehicle has entered an edge it needs to complete the distance, so congestion should be avoided before it enters the edge.

RETRACTED

TWM generator allows us to apply several routing policies: (a) apply *fixed weight penalty of value K* to the selected edges, or (b) apply a *random weight penalty amplified by value K* to the selected edges. Random distributions allow that different paths will be selected by the vehicles.

Algorithm 1 shows the ${\left[\mu_{k,m}\right]}_{x}$ generation process with $\Pi_{x}:{\left[\epsilon_{i,j}\right]}_{x},\left[\Omega_{k}\right],\left[\Gamma_{k,m}\right],R_{x}\to {\left[\mu_{k.m}\right]}_{x}$, where several data are required: the incidents location, the $\Pi_{x}$ function to use and its configuration parameters, and the radius distance $R_{x}$. TWM distribution follows these steps:

1. Obtain the TWM ${\left[\mu_{k,m}\right]}_{x}$ and set the time constraints $\left[\Gamma_{k,m}\right]$ on it. Sometimes it is not possible to know in advance the duration of the incident (as in traffic accidents) so it will be managed by means of monitoring.
2. Publish the TWM. Some of the fleets may not use it, as occurs with public transport using fixed routes.
3. Check time constraints:
  (a) If time constraints are known, disable TWM when they expire.
  (b) If they are unknown, monitor traffic conditions and disable TWM when they disappear.

**Algorithm 1**
$getTWMAroundEdge\left(\Theta ,\left[incident(name,lat,long)\right],\Pi_{lin}\left(k_{1},k_{2}\right)\right)\to {\left[\mu_{k,m}\right]}_{x}$
**Require:**
$\left[incident\left(name,lat,long\right)\right],\Theta ,\Pi_{lin}\left(k_{1},k_{2}\right),$
 1:$\left[\epsilon {}_{i,j}\right]\leftarrow readNetworkMap\left(\Theta \right)$
 2:${\left[\epsilon {}_{i,j}\right]}_{incident}\leftarrow locateIncidentEdges\left(\left[incident\left(name,lat,long\right)\right],\Theta \right)$
 3:**for all** $\epsilon {}_{k}\in {\left[\epsilon {}_{i,j}\right]}_{incident}$ **do**
 4:    ${\left[\epsilon {}_{i,j}\right]}_{TWM}\leftarrow getEdgesAroundRadius\left(\left[\epsilon {}_{i,j}\right],\epsilon {}_{k},R_{x}\right)$ 5:**end for** 6:**for all** $\epsilon {}_{k}\in {\left[\epsilon {}_{i,j}\right]}_{TWM}$ **do**
 7:    $tt_{i,j}\leftarrow getEdgeSpeed\left(\left[\epsilon {}_{i,j}\right],\epsilon {}_{k}\right)$ 8:    ${\left[\mu_{k,m}\right]}_{x}\left(\epsilon {}_{k}\right)\leftarrow \Pi_{lin}\left(tt_{i,j},k_{1},k_{2}\right)$ 9:**end for**


#### Incident Experiment Design

Traffic incidents have different impacts depending on traffic network usage. Any congestion control algorithm is not going to provide significant improvement in the case of low-congestion scenarios. We select an ad-hoc congested traffic scenario to analyze TWM impacts. It consists of a directional traffic flow of 2000 vehicles in one hour, which crosses the city from traffic assignment zones TAZ-5 and TAZ-50. These TAZs map to downtown dense populated neighborhoods. The network is congested in some points corresponding to edges in the best-route selection.The flow generates some congestion points in the most used edges.

RETRACTED

There is one traffic incident in a high occupation edge is shown in Figure 6, not being in one of the congested ones to avoid results skew. The incident occurs when the network starts to be heavily loaded, from time 2000 to 4800 s from a total simulation time of 7200 s (2 h).

A single ${\left[\mu_{1}\right]}_{x}$ TWM is used assuming that it is detected, generated, and distributed in the same time instant of the incident occurrence. The TWM is applied to all the fleets except for public transport (buses), which uses regular routes. The algorithm parameters used are:

- Impact radius $R_{x}=5$ selecting edges in a connected distance around the incident.
- Additive constant factor of 20 to discourage edge selection in radius, alpha factor of 5 to reinforce selection of edges in the best-route in case they are used $k_{1}=5,k_{2}=20$.
- Time constraints for incident duration $\Gamma_{k,m}\in \left[2000,4800\right]$.

### 5.7. TWM for Emergency Fleets

As a case study for fleet constraints, we designed a proof-of-concept (POC) scenario for emergency evacuations, where there is a specific area in a central point in the network (gas-station) that requires specific attention. There are three fleets considered: one standard traffic and two emergency fleets (firemen and policemen). The objective is that the emergency fleets run at free-flow in selected areas. Two emergency corridors must be established to the fire-station and the police-station as shown in Figure 7.

We use TWM to send specific maps to the vehicles over-weighting the emergency corridors in order to clear the standard traffic; less vehicles will use the path, only those that do require it. In the same way, a emergency map is created to force those vehicles related to the emergency to use the specific path. This study case differs from the ad-hoc incident management using a differential routing fulfilling specific requirements and constraints for emergency fleets.

Our POC experiment uses four TAZ areas as shown in Figure 8 with traffic flows crossing the city north–south and east–west. There are also additional emergency vehicles flows from/to the emergency area to the fire and police stations. Traffic has a uniform distribution with a 40 min duration and the simulation is executed over 60 min. Traffic flows are described in Table 8 showing vehicle payloads and the time range in minutes. We assume that 50% of the vehicles are using TWM.

RETRACTED

Our TWM now contains three maps: (1) $\mu_{F}$ for firemen routing inside their emergency corridor; (2) $\mu_{P}$ for policemen routing inside their emergency corridor; and (3) for the rest of the vehicles to discourage using the emergency corridors. $\mu_{F}$ and $\mu_{P}$ scale down original edge weights in the corridors, whilst $\mu_{V}$ adds weight penalty to these edges. Table 9 shows TWM parameters.

## 6. Results

Considering the case studies, we analyze the global impacts of TWM (travel-times, congestion, emissions, and pollution), and the impacts on the driving experience.

### 6.1. TWM Global Impacts

Several experiments are run over the city with the traffic demands explained and $\psi_{0.1}$, $\psi_{0.2}$, $\psi_{0.5}$, and $\psi_{1}$ driver adherences. We can see the impact of using TWM over travel-times in the histograms in Figure 9, which represent the travel-time distribution for all the trips. Table 10 compares the relative change of TWM usage over the non-TWM scenario considering different driver adherences. TWM usage reduces mean travel-times progressively with driver’s adoption, improving travel-time 19.6%. DTD, routed demand, also increases with TWM usage, up to 3.1%. Drivers are using alternative paths as TWM suggested, and this is the reason for this enhancement, but also for the slight mean route length increment (up to 1.9%).

Figure 10 shows total travel-times and total distances for all the vehicles where we can check that TTS has been significantly reduced (14%) and VKT suffers a 5% penalty as the drivers use routes different from the best-cost physical route.

Figure 11 shows how the rest of global variables evolves in time comparing increasing driver adherences to TWM: edge congestion (NEO(C)) is reduced, mean network speed (NMS) increases and number of congested vehicles (NMV(H)) is reduced. A positive driving experience when using TWM encourages new adherences to grow in next traffic cycles.

We can observe in Figure 12 left heat-map of the network at timestamp 3000 showing density of halted vehicles and top-used edges. This data may be used for MuTraff feedback and create historical records to create TWM routing based on historical data. This TWM may discourage selecting these edges for the best-routes.

#### 6.1.1. TWM Impact on User Driving Experience

Driver’s adherence to TWM is a critical factor for success and improvement. It is achieved by means of three main streams: individual perception that enables viral word-of-mouth adoption, marketing campaigns, and/or legal recommendations or constraints. Individual perception is usually measured by the NPS key performance indicator (net promoting score) that compares promoters and detractors when asked for the individual recommendation based on own experience [78].

RETRACTED

Global statistics mask individual perceptions and it makes necessary to compare each single trip under TWM and non-TWM scenarios. Histograms of individual travel-times improvement $TTC_{rel}$ help us to analyze this factor showing how many drivers have been negatively or positively impacted. Real adoption models of TWM should combine both objective factors (route length, travel-time, and cost) and subjective factors (halted-times, crossings, etc). Figure 13 shows $TTC_{rel}$ for $\psi_{0.5}$ and $\psi_{1}$ adherences. It shows the objective improvement at the right side of both diagrams: A large number of drivers have significantly reduced their travel-times with respect to the original travel-times. They were the previously congested vehicles.

TWM benefits reach all the vehicles, not only to those that use TWM. This is the obvious consequence of routing some traffic out of the shortest paths: The whole network status gets improved.

Figure 14 shows the cumulative probability distribution for travel-time improvement at $\psi_{0.1}$, $\psi_{0.2}$, $\psi_{0.5}$ and $\psi_{1}$ adherences. Even at very low adoption scenarios such as $\psi_{0.1}$ (10%) the probability of being positively impacted is remarkable. TWM provides early global impacts even with a small volume of drivers.

#### 6.1.2. Comparison of Benefits for TWM and Non-TWM Users

Under normal situations, the traffic network holds TWM and non-TWM users. Traffic variations affect both of them. Figure 15 details two overlapped histograms considering adherences of $\psi_{0.2}$ and $\psi_{0.5}$. In the first scenario, the positive slope shows that non-TWM users are being highly improved in their travel-time perception by the TWM users. For $\psi_{0.5}$ we see that both populations are obtaining similar benefits. TWM drivers are using alternative TWM best-routes considering new network views, and then clearing edge occupation in the non-TWM best-routes. We call it the TWM route clearing effect.

#### 6.1.3. TWM Impacts on Pollution Emissions

Figure 16 shows that TWM with random maps has a remarkable impact on all the global emission parameters $GET_{NOx,CO,CO2,HC,PMx}$ reducing them up to 12%. Fuel consumption $PCT_{Fuel}$ is reduced by 7.5%. Noise footprint is also improved by 4.3%.

In spite of these improvements, global metrics in this urban topology are affected by the large routing capacity of the highways in the traffic network that route a large part of the vehicles. We should consider the situation in dense-populated neighborhood with no highways affection. In Figure 17 we have selected a dense-populated area to analyze how pollution has been affected by TWM. Even with very low adherences ( $\psi_{0.1}$) pollution is reduced very significantly reaching 18% in case of $GET_{PMx}$. As we increase TWM adoption, we reach up to 40% reduction. The noise footprint is also reduced in a similar way. Individual traffic is best routed by alternative paths.

RETRACTED

### 6.2. Dynamic Incident Management

Several driver adherences of $\psi_{0.1}$, $\psi_{0.2}$, $\psi_{0.5}$, and $\psi_{1}$ are considered for multimap adoption experiments.

Figure 18 and Table 11 show TWM ${\left[\mu_{1}\right]}_{x}$ impacts for $\psi_{0.5}$ and $\psi_{1}$ adherences. TWM clears congestion suggesting best-route alternatives considering over-weighted edges around the incident. Travel-time variation perceived by the drivers in this case raises up to 52% for a full $\psi_{1}$ adherence, though it depends on concrete scenario: road network, time-instant, traffic payload, and other factors. Histograms compare the same incident scenario using TWM under two different adherences (0.5 and 1.0; in red) and the non-TWM situation (green). Congestion peaks occur at the right side (green) and progressively cleared with TWM usage (red).

Figure 19 shows the incident impact on global congestion, raising the number of halted vehicles in the network. It also shows the impact of ${\left[\mu_{1}\right]}_{x}$ TWM with different adherences on halted vehicles NMV(H), on congested edges NEO(C) and in network mean speed NMS. As the adherence increases, best results are obtained, leading even to full congestion mitigation.

Subjective individual variation is shown in Figure 20 for $\psi_{1}$ adherence where it is clear that vehicles that where initially blocked by the incident (right-side) have obtained a great reward for using TWM in terms of travel-time. Very few vehicles have been negatively impacted.

Figure 21 shows that global gas emissions $GET_{NOx,CO,CO2,HC,PMx}$ are reduced in the same rate as the incident is cleared, always depending on the number of TWM adopters for the clearing map. Also noise emissions are reduced, though $\psi_{1}$ adherence reverses the situation as vehicles run at higher speed increasing noise.

### 6.3. TWM for Emergency Fleets

Figure 22 and Figure 23 represent the same timestamp in the scenarios of no-TWM and TWM with 50% adherence application. In Figure 22 standard traffic uses the whole network together with the emergency fleets (firemen and policemen). In Figure 23 TWM application has cleared the two emergency corridors, routing standard traffic to alternative paths. Fire and police vehicles run at free-flow speeds, having a low travel-time variance (<1%).

RETRACTED

## 7. Conclusions and Future Work

Traffic weighted multimaps is a traffic routing mechanism that focuses on multi-objective traffic routing needs. TWM maps are generated for the different traffic groups. TWM relies on big-data usage and enables static and dynamic traffic management and can be used for a wide range of scenarios, from global concerns to spurious incidents. Some of which were shown in this paper, i.e., global congestion management and dynamic incident management. Also, experiments show how individual driving experience is perceived in relationship to TWM adoption models. MuTraff architecture has been introduced as a feasible technical platform that can be seamlessly integrated into existing planning and routing platforms and also existing traffic agents.

The experiments have used a real urban traffic network under real traffic conditions, to show how MuTraff can provide TWM-based solutions that improve all the global indicators: travel-time reduction, congestion reduction (halted vehicles, congested edges, and others), pollution gas emissions, and noise footprints.

Simplicity, scalability, and safety have a cost. TWM is a stochastic routing technique that has not been designed to achieve theoretical optimal solutions as in other centralized routing solutions. Thus, there is plenty of research to be done to design more advanced algorithms to calculate TWM maps and improve routing. The stochastic nature of TWM and the use of random maps do not guarantee to improve travel time for all the vehicles in the network. We need to implement new algorithms to generate maps in specific scenarios: congestion avoidance, evacuation, contingency plans, etc. In our work we are not considering driver behavior from a temporal perspective, which may have a strong influence on the adoption of TWM. This issue requires system dynamics analysis in order to study TWM adoption, where improved and penalized vehicles modulate a feedback loop that will affect the adoption rate. In relation to drivers’ behavior during the travel-time, we have not considered the influence of rerouting according to current traffic conditions.

The improvement achieved by TWM depends mainly on: (a) scenario conditions, (b) adherence of traffic agents to TWM, and (c) design of the $\Pi_{x}$ optimization function to cope with congestion situations. TWM has limited impact in low-traffic scenarios, as agents are close to their ideal performance (travel-time), though in all situations network and fleet performance indicators are improved. TWM offers its best performance capabilities in high-density traffic scenarios and congestion, enhancing individual objectives and also improving group and global indicators. Real-time response to network and traffic incidents is fast and effective, and TWM is able to release new ad-hoc multimaps for a new situation using the available information.

RETRACTED

The benefits of MuTraff for TWM management include: (a) usage of big-data techniques to handle complex traffic scenarios and control policies where analytical solutions require heavy computing to get optimal solutions; MuTraff provides a fast response pseudo-optimal solution; (b) it offers an early and real-time decision making environment for drivers and traffic authorities; (c) it is conceived as a modular platform based on standard open-source frameworks and is able to evolve rapidly in the future; (d) it offers back-end services for route planning and also REST-APIs for route calculation at agent side, compatible with most of the existing traffic platforms; (e) MuTraff preserves traffic agents autonomy as TWM takes into account individual freedom of route choice; (f) MuTraff preserves data privacy: no individual identification or tracking is required; and (g) it works with partial adoption models as it does not require that all the vehicles use it. It may be used in a biased manner (only for certain categories or policies).

TWM contributes to innovation with a practical and feasible proposal as shown with MuTraff architecture, enabling a big-data based model suitable for application in the broader concept of smart cities. It allows multi-objective management of needs from different traffic categories: standard traffic, public transportation, electric vehicle, pay-to-drive and car-sharing fleets, commercial distribution, disabled people, pollutants, dangerous transport, routing due to weather, timetables, etc. It is self-replenished and self-learning. MuTraff and TWM may be used with standard optimization algorithms and techniques for route calculation. They do not require V2V communications nor specific sensors or signaling, and the computing infrastructure required may be allocated in a cloud with elastic capabilities.

There are many future research possibilities that have been pointed out in the paper: (a) creating optimal static TWM distributions for historical data with evolutionary algorithms, (b) creating dynamic traffic assignment models using TWM based on previous driver experiences as we have shown that they may be critical for TWM adherence, (c) using TWM for zone routing policies as pointed by [49], (d) applying TWM to hyperpath calculation using techniques described by [12,34], (e) creating evolutionary algorithms and optimization functions for finding local area minimum for routing maps that can cover eventual time-dependent situations, and (f) extension of the MuTraff MTS simulator with mesoscopic simulation engines.

RETRACTED

## Figures and Tables

**Figure 1:** Multimap traffic control architecture (MuTraff) architecture blocks. MuTraff simulator (MTS), MuTraff big-data core (MDB), MuTraff central control station (MCCS), MuTraff traffic and maps toolbox (MTools).

**Figure 2:** MuTraff components detailed.

**Figure 3:** MuTraff simulator (MTS) main loop and SUMO integration.

**Figure 4:** Alcala de Henares traffic network and TAZ mapping.

**Figure 5:** Alcala crowdsensing data (position and real speed), October 2019. Courtesy of www.satya-insights.com.

**Figure 6:** Incident in the main traffic flow and radius 5 TWM response.

**Figure 7:** Emergency corridors for police and firemen.

**Figure 8:** Synthetic traffic flows for emergency simulation.

**Figure 9:** Alcala de Henares, TWM impact on travel-time with $\psi_{0.5}$ and $\psi_{1}$ adherences.

**Figure 10:** Total travel-time (TTS) and total distance (VKT).

**Figure 11:** Congested edges (NEO(C)), network speed (NMS) and halted vehicles (NMV(H)) at $\psi_{0}$, $\psi_{0.2}$, $\psi_{0.5}$ and $\psi_{1}$ adherences.

**Figure 12:** Congestion traffic experiments in Alcala de Henares, halted vehicles and most congested edges.

**Figure 13:** Individual travel-time experience $TTC_{rel}$ at $\psi_{0.5}$ and $\psi_{1}$ adherences.

**Figure 14:** Cumulative probability distribution for travel-time improvement at $\psi_{0.1}$, $\psi_{0.2}$, $\psi_{0.5}$, and $\psi_{1}$ adherences.

**Figure 15:** TWM and non-TWM travel-time improvement for $\psi_{0.2}$ and $\psi_{0.5}$ adherences.

**Figure 16:** Global effects on gas emissions $GET_{NOx,CO,CO2,HC,PMx}$, energy consumption $PCT_{Fuel}$ and noise emissions NET using 16-TWM at $\psi_{0}$, $\psi_{0.2}$, $\psi_{0.5}$, and $\psi_{1}$ adherences.

**Figure 17:** Local effects (Barrio Juan de Austria) on gas emissions $GET_{NOx,CO,CO2,HC,PMx}$, energy consumption *$PCT_{Fuel}$,* and noise emissions NET using 16-TWM at $\psi_{0.1}$, $\psi_{0.2}$, $\psi_{0.5}$, and $\psi_{1}$ adherences.

**Figure 18:** Travel-time variation with ad-hoc TWM on incident for $\psi_{0.5}$ and $\psi_{1}$.

**Figure 19:** Incident impact without TWM and effect of TWM on halted vehicles NMV(H), congested Edges NEO(C), and network speed NMS.

**Figure 20:** Individual travel-time relative variation.

**Figure 21:** Effects on pollutants emissions $GET_{NOx,CO,CO2,HC,PMx}$, energy consumption $PCT_{Fuel}$ and noise emissions NET during incident clearing using TWM.

RETRACTED

**Figure 22:** Traffic intensity at minute 42. No TWM.

**Figure 23:** Traffic intensity at minute 42. TWM with 50% adherence.

**Table 1:** Model summary. Traffic weighted multimaps (TWM).

ID	Description	ID	Description
Θ	Urban network representation.	$\left[\mu_{k,m}\right]$	TWM multimap. *m* = number of maps per fleet.
Φ	Traffic density data	$\mu_{k,m}$	Single map instance for vehicle group $\Omega_{k}$
$\eta_{n}$	Traffic network node	Π	TWM weight evaluation function.
$\epsilon_{i,j}$	Edge connecting nodes $\eta_{i}$ and $\eta_{j}$.	$\Pi_{std}$	Standard map weight evaluation function.
$d_{i,j}$	Length of edge $\epsilon_{i,j}$.	$\Pi_{\delta }$	TWM weight function based on random distributions.
$S_{i,j}$	Max speed allowed for edge $\epsilon_{i,j}$.	$\Gamma_{k,m}$	Time constraints for map $\mu_{k,m}$.
$tt_{i,j}$	Min travel-time for edge $\epsilon_{i,j}$, $tt_{i,j}=\frac{d_{i,j}}{S_{i,j}}$	*⨙*	Routing algorithm: Dijkstra, A*, etc.
$\Delta_{m}$	TAZ, traffic assignment zone.	$\psi_{k}$	TWM adherence factor of fleet $\Omega_{k}$.
$\Omega_{k}$	Vehicle group (fleet). *k* = number of groups	$R_{a}^{k,m}$	Route selected by vehicle $\upsilon_{a}^{k}$ for trip $W_{a}^{k}$ using $\mu_{k,m}$.
$\Omega_{0}$	Default generic vehicle group.	$RL_{a}^{k}$	Route length of $R_{a}^{k,m}$.
$\left[\upsilon_{a}^{k}\right]$	Vehicle population. Vehicles are $\upsilon_{a}^{k}$.	$TT_{a}^{k}$	travel-time of $R_{a}^{k,m}$.
$W_{a}^{k}$	Individual trip of $\upsilon_{a}^{k}$ from origin $O_{a}$ to destination $D_{a}.$	$STT_{a}^{k}$	Total congested time of $R_{a}^{k,m}$.
$\left[P_{a}^{k}\right]$	Sets of planned stops for the trip $W_{a}^{k}$.	$MTT_{a}^{k}$	Total non-congested time of $R_{a}^{k,m}$.

**Table 2:** Traffic fleet composition.

Fleet	%	Traffic Mix	Use TWM	Emissions
Car	50%	random + directional	Yes	HBEFA3/PC_G_EU4
Taxi	20%	random + directional	Yes	HBEFA3/PC_G_EU4
Bus	10%	random + directional	No	HBEFA3/LAV_D_EU4
Motorcycle	20%	random + directional	Yes	HBEFA3/LDV_G_EU6

**Table 3:** Driver adherence.

Confidence	Value
Small confidence	10%
Mid confidence	20%
Big confidence	50%
Full adoption	100%

**Table 4:** TWM indicators summary.

Indicator	Description	Indicator	Description
DTD	Ratio of completed traffic demand.	$NEO^{t}$	Instant network edge occupancy.
$DTD_{TWM}$	Ratio of completed traffic demand using TWM.	$GET_{NOx,CO,CO2,HC,PMx...}^{t}$	Instant total pollutant emissions.
TTS	Total travel-time.	$NET^{t}$	Instant total noise emissions.
THS	Total halted travel-time.	$PCT_{Fuel,Electricity}^{t}$	Instant total power consumption.
NHD	Halted demand of vehicles (speed < 0.1 m/s).	$TTC_{a}^{k}$	Individual travel-time improvement when using TWM.
VKT	Total routed distance.	$RLC_{a}^{k}$	Individual trip-length improvement when using TWM.
$NMS^{t}$	Instant network mean speed.	$MR_{a}^{k}$	Individual motion rate, percentage of travel-time not halted.
$NMV^{t}$	Instant routing vehicle volume.		

RETRACTED

**Table 5:** TAZ description and usage.

TAZ	Type	Name	Description	Main Usages
TAZ-1	Highway	E-5, N-2 West	Main National Highway, Madrid–Barcelona.	Crossing traffic, work trips, logistics
TAZ-2	Highway	E-5, N-2 East	Main National Highway, Madrid–Barcelona.	Crossing traffic, work trips, logistics
TAZ-3	Highway	M-100 South–West	Regional Highway (Mejorada)	Crossing traffic, work trips, logistics
TAZ-4	Highway	M-100 North	Regional Highway (Daganzo)	Crossing traffic, work trips, logistics
TAZ-5	Road	M-300 West	Regional Road (Alcala)	Crossing traffic, work trips, logistics
TAZ-6	Road	M-300 South	Regional Road (Loeches)	Crossing traffic, work trips, logistics
TAZ-7	Road	M-119 North	Regional Road (Camarma)	Crossing traffic, work trips, logistics
TAZ-8	Road	M-121 North	Regional Road (Meco)	Crossing traffic, work trips, logistics
TAZ-50	Area	La Dehesa/Cuadernillos	Commercial Area North–East	Commercial and Distribution
TAZ-51	Area	La Garena	Commercial Area West	Commercial and Distribution
TAZ-60	Area	Universidad	University campus, Hospital, Research industries	Services, public transports
TAZ-70	Area	Paracuellos, Daganzo	Industrial Estate	Industry and Logistics
TAZ-71	Area	La Garena	Industrial Estate	Industry and Logistics
TAZ-90	Area	City Center	Population	Standard trips and public transports
TAZ-91	Area	Espartales	Population	Standard trips and public transports

**Table 6:** Traffic demands per O/D TAZ.

TAZ Num.	TAZ-90	TAZ-91	TAZ-1	TAZ-2	TAZ-3	TAZ-4	TAZ-5	TAZ-6	TAZ-7	TAZ-8	TAZ-50	TAZ-51	TAZ-60	TAZ-70	TAZ-71
**TAZ-90**	8000	200	800	800	400	400	1000	400	400	400	200	200	200	100	100
**TAZ-91**	200	100	300	300	150	150	100	100	100	100	100	100	100	50	50
**TAZ-1**	800	500		2000							100	100	200	200	200
**TAZ-2**	800	500	2000								100	100	200	200	200
**TAZ-3**	400	100	400	400		1000					100	100	100	50	50
**TAZ-4**	400	100	400	200	1000						100	100	100	50	50
**TAZ-5**	800	100						400			100	100	100	50	50
**TAZ-6**	800	100		400			1000				100	100	100	50	50
**TAZ-7**	400	100	300	100							100	100	100	50	50
**TAZ-8**	400	100	300	100							100	100	100	50	50
**TAZ-50**	200	100	100	100	100	100	100	100	100						
**TAZ-51**	200	100	100	100	100	100	100	100	100						
**TAZ-60**	200	50	200	200	100	100	100	100	100					50	50
**TAZ-70**	100	50	200	200	50	50	50	50	50	50			50		
**TAZ-71**	100	50	200	200	50	50	50	50	50	50			50		

**Table 7:** TWM fleet usage.

Fleet	$\mu_{0}$	$\mu_{1}$	$\mu_{2}$	$\mu_{3}$	...	$\mu_{16}$
Bus	1.0	0	0	0	...	0
Car	0	0.063	0.063	0.063	...	0.063
Taxi	0	0.063	0.063	0.063	...	0.063
Motorcycle	0	0.063	0.063	0.063	...	0.063
Truck	0	0.063	0.063	0.063	...	0.063
Trailer	0	0.063	0.063	0.063	...	0.063

RETRACTED

**Table 8:** Emergency traffic flows, showing volume and time span (from-to min).

From/To	North TAZ	South TAZ	East TAZ	West TAZ	Police St.	Fire St.	Emergency Area
**North TAZ**		500 [0–40]					
**South TAZ**	500 [0–40]						
**East TAZ**				500 [0–40]			
**West TAZ**			500 [0–40]				
**Police St.**							50 [10–40]
**Fire St.**							50 [10–40]
**Emergency Area**					50 [25–40]	50 [25–40]	

**Table 9:** TWM configuration.

Parameter	$\mu_{V}$	$\mu_{F}$	$\mu_{P}$
**Map name**	Vehicles on emergency	Firemen	Policemen
**Adherence**	50% except emergencies	100% Firemen	100% Policemen
**Edges Affected**	Emergency corridor	Emergency corridor	Emergency corridor
**Fleet policy**	Any, except emerg.corridor	Free flow	Free flow
**Weight Policy**	Penalty	Reduction	Reduction
**Impact Radius**	1	1	1
**$k_{1}$**	5	0,1	0,1
**$k_{2}$**	10	0	0
**From/to time**	[10–40]	[10–40]	[10–40]

**Table 10:** Alcala de Henares, TWM impact with $\psi_{0.1}$, $\psi_{0.2}$, $\psi_{0.5}$ and $\psi_{1}$ adherences.

16 Maps-Uniform05		No TWM	10%	20%	50%	100%
Traffic	Demand	18,694	18,694	18,694	18,694	18,694
	Using TWM	0	1846	3731	9385	18,694
	Routed	17,895	17,667	18,067	18,042	18,447
	% Routed, DTD	-	−1.27%	0.96%	0.9%	3.08%
Travel-time TT	Mean		−3.41%	−4.75%	−9.17%	−19.60%
Route Length RL	Mean		1.10%	0.73%	1.59%	1.90%

**Table 11:** TWM impact on travel-time at incident scenario for $\psi_{0.5}$ and $\psi_{1}$.

Incident, + 1 TWM, $\left[\mu_{1}\right],\Pi_{\mathrm{lin}}\left(k_{1}=5,k_{2}=20\right)$		No TWM	50%	100%
Traffic	Demand	500	500	500
	Using TWM	0	241	500
	Routed	500	500	500
Travel-time	Mean		−32.67%	−52.36%
Route Length	Mean		−0.10%	−1.04%

## Abbreviations

The following abbreviations are used in this manuscript:

DWM	MuTraff Middleware
GPS	Global Positioning System
HBEFA	The Handbook Emission Factors for Road Transport (HBEFA)
ITS	Intelligent Transportation Systems
MCCS	MuTraff Central Control Station (subsystem)
MDB	MuTraff Big-Data Subsystem (subsystem)
MTA	MuTraff Mobile Agents (subsystem)
MTools	MuTraff Auxiliary Toolkit
MTS	MuTraff Traffic Simulator
MuTraff	System Architecture for TWM
OSM	OpenStreet Maps
SAN	Sensor and Actuator
SUMO	Simulation for Urban Mobility
TMS	Traffic Management System
TWM	Traffic Weighted multimaps
UAH	Universidad de Alcala
XML	eXtensible Markup Language
